# Molecular Mechanisms of *Gynostemma pentaphyllum* in Prevention and Treatment of Non-Small-Cell Lung Cancer

**DOI:** 10.1155/2022/9938936

**Published:** 2022-09-06

**Authors:** Renji Liang, Jinzheng Wu, Ronghua Lin, Liling Ran, Bo Shu, Hao Deng

**Affiliations:** ^1^Department of Cardiothoracic Surgery, The First Affiliated Hospital, Hengyang Medical School, University of South China, Hengyang 421001, China; ^2^Department of Anesthesiology, The Second Xiangya Hospital, Central South University, Changsha 410011, China; ^3^Department of General Surgery, Huichang County People's Hospital, Huichang 342600, Jiangxi, China; ^4^Hunan Aerospace Tianlu Advanced Material Testing Co., Ltd., Changsha 410000, China; ^5^Department of General Surgery, The Second Xiangya Hospital, Central South University, Changsha 410011, Hunan, China

## Abstract

**Objective:**

Lung cancer represents the leading cause of cancer death on a global scale. *Gynostemma pentaphyllum* (*G. pentaphyllum*), a traditional medicinal material with a high medicinal and health value, has recently been reported for its anticancer activity. However, the pharmacological mechanism of *G. pentaphyllum* in non-small-cell lung cancer (NSCLC) remains to be elucidated.

**Methods:**

The active ingredients of *G. pentaphyllum* were obtained from the TCMSP database and known therapeutic targets of NSCLC from the GeneCards and OMIM databases. Disease-drug common targets are subjected to protein-protein interaction (PPI), GO enrichment analysis, and KEGG pathway enrichment analysis. A molecular docking strategy was performed to verify the interaction between molecules.

**Results:**

We found a total of 24 compounds of *G. pentaphyllum* fulfilling OB ≥ 30% concomitant with DL ≥ 0.18 and corresponding 81 target genes in the TCMSP database, with 5062 NSCLC-related genes collected in the GeneCards and OMIM databases. The network consisting of the disease-target compound was obtained, including 8 active ingredients and 69 common targets. The PPI network with 65 nodes and 645 edges was visualized. After functional enrichment analysis, it was revealed that the therapeutic effects of *G. pentaphyllum* on NSCLC were achieved through response to ketone, gland development, and cellular response to xenobiotic stimulus. After molecular docking analysis, it was revealed that the two active ingredients of *G. pentaphyllum,* quercetin and rhamnazin, bound well and stably to their targets (MYC, ESR1, and HIF1A).

**Conclusion:**

Our study, based on network pharmacology, identifies active ingredients, targets, and pathways model mechanism of *G. pentaphyllum* when it is used to treat NSCLC.

## 1. Introduction

In spite of remarkable progress in understanding of pathogenesis, application of predictive biomarkers, immunologic control, and therapeutic strategies for lung cancer in the past two decades, lung cancer still contributes to a heavy global burden of cancer mortality and morbidity, with an estimated 2 million new diagnoses and 1.76 million deaths each year [1]. Although the male-to-female ratio differs across regions, higher incidence and death rates of lung cancer (roughly 2 times) have been estimated in men than in women on the whole [2]. Lung cancer is a heterogeneous disease that consists of various histological and molecular types with clinical relevance, and the vast majority of patients (accounting for roughly 85%) are afflicted by non-small-cell lung cancer (NSCLC). Surgical care for early-stage NSCLC has been developed with new procedures, techniques, and care pathways [3]. When patients are diagnosed with NSCLC, locally advanced but surgically resectable, the optimal treatment includes at least radiochemotherapy. With regard to those with unresectable or inoperable locally advanced disease, radiochemotherapy followed by immunotherapy consolidation has evolved as a new standard of care [4]. Over the past two decades, a proportion of NSCLC patients have experienced long-term clinical benefits from molecular targeted therapies and immunotherapies, but acquired resistance to current treatments during treatment or after treatment is still a clinical challenge [5, 6].

Emerging studies with experimental models have proved therapeutic effects of herbal medicines on several common human cancers including NSCLC [7, 8]. *Gynostemma pentaphyllum* (*G. pentaphyllum*) is a creeping perennial herb that is sourced from the family Cucurbitaceae, which is widely used as a herbal medicine and distributed in Asian regions, especially in China [9]. *G. pentaphyllum* was first recorded as Traditional Chinese Medicine (TMC) in *Jiuhuang Bencao,* written by Zhu Su, who was a Chinese botanist in AD 1406 [10]. The anticancer activity [11], antiobesity effect [12], antioxidant and anti-inflammatory effects [13], and antifibrotic effect [14] of the main active ingredients of *G. pentaphyllum* have been widely reported.

TMC has several characteristics, such as multicomponent and multitarget synergistic effects, while it is difficult to systematically and comprehensively detect the exact mechanism of TMC through traditional methods. Network pharmacology is a novel approach that was proposed by Hopkins in 2008 to study the molecular mechanisms of drug action, for example, natural herbs and TCM, by establishing computer-aided networks on the basis of “multigene,” “multitarget,” and “multichannel” linking with multiple compounds [15]. In addition, molecular docking verification is performed to estimate the binding energy between TCM components and disease targets and to explain how ligands act on complex molecular networks. In this work, we aim to elucidate the therapeutic mechanism of *G. pentaphyllum* for NSCLC based on network pharmacology followed by molecular docking analysis.

## 2. Methods

### 2.1. Active Ingredients and Putative Target Genes of *G. pentaphyllum*

To obtain the active ingredients of *G. pentaphyllum*, we performed a computer-based retrieval in the Traditional Chinese Medicine Systems Pharmacology Database and Analysis Platform (TCMSP, https://lsp.nwu.edu.cn/tcmsp.php), which is a popular pharmacology database where there are almost 500 formulae of TCM concomitant with 30,069 compounds. Two pharmacokinetic parameters related to ADME (absorption, distribution, metabolism, and excretion), oral bioavailability (OB), and drug-likeness (DL), were evaluated to retain the active ingredients of *G. pentaphyllum* for further investigation. In this study, the active ingredients of *G. pentaphyllum* must fulfill OB ≥ 30% and DL ≥ 0.18. The protein targets of the active ingredients were also predicted in the TCMSP database, with the gene names obtained from the UniProt Knowledgebase (UniProtKB), which collects functional information on proteins covering accurate, consistent, and rich annotation.

### 2.2. Common Target Genes of NSCLC and *G. pentaphyllum*

The known therapeutic targets of NSCLC were dug up in the GeneCards combined database with the Online Mendelian Inheritance in Man database (OMIM, https://omim.org/). The proteins (only “*Homo sapiens*”) associated with NSCLC were chosen. Using the Venn functional intersection in the *R* software, overlapping targets of *G. pentaphyllum* and NSCLC were obtained.

### 2.3. Protein-Protein Interaction (PPI) Network Construction

The common targets of *G. pentaphyllum* and NSCLC were entered into the STRING database (https://www.string-db.org/) to estimate their PPIs. The species should be “*Homo sapiens*” and the confidence score should be no less than 0.4. The PPI network was visualized by importing the TSV-based file to Cytoscape software (3.8.1). According to the degree value obtained using the cytoHubba plug-in of Cytoscape, the key genes were extracted.

### 2.4. Functional Enrichment Analysis

The disease-drug overlapping targets of *G. pentaphyllum* and NSCLC were subject to Gene Ontology (GO) and Kyoto Encyclopedia of Genes and Genomes (KEGG) enrichment analyses using the “clusterProfiler” package in R/Bioconductor. We mapped them into the DAVID Bioinformatics Resources 6.7 (https://david-d.ncifcrf.gov/), with the species set as “*Homo sapiens*” and *P* value < 0.05 set as a cutoff value. Results of GO analysis were visualized using the OmicShare platform (https://www.omicshare.com/), focusing on three levels: biological process (BP) analysis, cellular component (CC) analysis, and molecular function (MF) analysis.

### 2.5. Molecular Docking Verification

The protein ligand complexes of targets with high-ranking degree values in the PPI network were obtained using the RCSB database (https://www.rcsb.org/). The molecular docking verification was performed on the Systems Dock Website (https://systemsdock.unit.oist.jp/iddp/home/index) to evaluate the binding strength and activity between those protein ligand complexes and the active ingredients of *G. pentaphyllum*, with core chemical compounds sorted out.

## 3. Results

### 3.1. The Active Ingredients of *G. pentaphyllum*

When searching the active ingredients of *G. pentaphyllum* and set OB ≥ 30% concomitant with DL ≥ 0.18 in the TCMSP database, we found a total of 24 compounds of *G. pentaphyllum* (Table 1), including 3′-methyleriodictyol, rhamnazin, sitosterol, ruvoside_qt, spinasterol, campesterol, isofucosterol, ginsenoside f2, CLR, quercetin, (24S)-Ethylcholesta-5,22,25-trans-3beta-ol, 4*α*,14*α*-dimethyl-5*α*-ergosta-7,9(11),24(28)-trien-3*β*-ol, cucurbita-5,24-dienol, cyclobuxine, and 10 from gypenoside.

### 3.2. Identification of Disease-Drug Common Targets

After removal of duplicate values and conversion of protein names into gene symbols, we obtained 81 target genes of the active ingredients of *G. pentaphyllum* in the TCMSP database. Subsequently, we searched for known therapeutic targets of NSCLC in authoritative open databases and obtained 4861 and 201 targets in the GeneCards and OMIM databases, respectively. After the removal of duplicate values, 4970 therapeutic targets of NSCLC were obtained. Venn intersection analysis by *R* software showed there were 69 overlapping target genes of NSCLC and *G. pentaphyllum* (Figure 1). We then used Cytoscape software to visualize the disease-target-compound network, which consisted of 8 active ingredients and 69 common targets (Figure 2). The 8 bioactive compounds included *3′-methyleriodictyol* (1 node), *rhamnazin* (9 nodes), *sitosterol* (2 nodes), *spinasterol* (16 nodes), *campesterol* (1 node), *isofucosterol* (16 nodes), *CLR* (2 nodes), and *quercetin* (107 nodes).

### 3.3. PPI Network Construction

We imported 69 common targets between NSCLC and the active ingredients of *G. pentaphyllum* into the STRING database. As shown by Figure 3(a), there were 65 nodes with 645 edges of the PPI network where higher degree values reflecting closer correlation (Figure 3(b)), and PRSS1, EIF6, RUNX1T1, and NPEPPS were removed due to weak interaction.

### 3.4. Enrichment Analysis for Disease-Drug Common Targets

Next, we conducted GO annotation and KEGG pathway analyses of 69 disease-drug common targets. After GO analysis, we found 1211 GO terms were significantly enriched by these disease-drug common targets (Figure 4(a), *p* < 0.05). At the level of BP, the active ingredients of *G. pentaphyllum* were associated with 1106 terms. At the level of CC, the active ingredients of *G. pentaphyllum* were associated with 11 terms. At the level of MF, the active ingredients of *G. pentaphyllum* were associated with 94 terms. After KEGG pathway analysis, we found 11 KEGG pathways were significantly enriched by these disease-drug common targets (Figure 4(b), *p* < 0.05).

### 3.5. Molecular Docking Verification

For the sake of estimating the interaction between ligand and receptor and to assess the binding mode and affinity according to theircomprehensive characteristics, a molecular docking strategy was performed by the AutoDockTools. Three candidate targets, MYC, ESR1, and HIF1A, were selected for molecular docking analysis according to higher degree values in the core PPI network. The binding energy less than 0 indicates spontaneous binding of ligand and receptor, and smaller values reflect higher binding activity. The affinity energy ≤ −5 kcal/mol is considered high affinity. It was found that the binding energy of quercetin and MYC was −8.50 kcal/mol, rhamnazin and ESR1 was −8.40 kcal/mol, quercetin and HIF1A was −8.90 kcal/mol, suggesting that the 2 potential active compounds of *G. pentaphyllum*, quercetin and rhamnazin, have good binding ability with the targets MYC, ESR1, and HIF1A (Figure 5).

## 4. Discussion

TCM theory believes that the basic pathogenesis of lung cancer is attributed to the deficiency of the body's Yuan Qi with the excessiveness of pathological products (phlegm-blood stasis syndrome) within the human body and that “invigorating Qi for consolidation of the exterior” is an effective way to treat lung cancer [16]. With the substantial advancements in modern medicine, the mechanisms behind the therapeutic implications of TCM in lung cancer are involved in improving the body's immune function, inducing tumor cell apoptosis, and preventing tumor angiogenesis [17]. The active ingredients of *G. pentaphyllum* have been studied for their characteristics of clearing away heat and toxic materials, replenishing Qi and invigorating the spleen, and lung-moistening phlegm-transforming, which can be used to fight the basic pathogenesis of lung cancer [18–20]. Nevertheless, it is still a clinical challenge for the clinical translation of *G. pentaphyllum* for NSCLC treatment considering the complexity of the active ingredients and multiple targets of *G. pentaphyllum*. In the beginning, we searched the TCMSP database to collect putative molecules of *G. pentaphyllum* compounds and then searched the GeneCards and OMIM databases to collect therapeutic targets of NSCLC. Disease and drug common targets were acquired by Venn intersection and subjected to PPI analysis by functional enrichment analysis. The best binding mode of CS compounds and common target proteins was evaluated by molecular docking and analysis in AutoDockTools. In this work, the authors, with the help of a network pharmacology approach followed by molecular docking verification, attempt to elucidate the pharmacological mechanism of *G. pentaphyllum* on NSCLC treatment.

In the system of TCM, compounds fail to be delivered to the target organs to produce biological activities due to a lack of proper pharmacokinetic properties [21]. The network pharmacology approach integrates information from biological systems, drugs, and diseases, providing a systemic analysis of the pharmacokinetic properties of TCM. Usually, 30% of OB concomitant with 0.18 of DL was the lowest level to evaluate the pharmacokinetic actions of the compounds of herbal medicines. In our disease-target-compound network, 8 bioactive compounds in *G. pentaphyllum* stood out, which may responsible for the leading therapeutic effects of *G. pentaphyllum* on NSCLC, including *3′-methyleriodictyol*, *rhamnazin*, *sitosterol*, *spinasterol*, *campesterol*, *isofucosterol*, *CLR*, and *quercetin*. *Quercetin* ranked the highest with 107 targets of NSCLC, followed by the other three bioactive compounds, *isofucosterol*, *spinasterol*, and *rhamnazin*. *Quercetin* has a variety of biological properties, such as antioxidant, anti-inflammatory, and antiapoptosis [22–24], which has been widely investigated in human cancers, including lung cancer. It was reported that the antiproliferative effects on lung cancer cells by caspase-dependent DNA damage signaling [25]. More profoundly, Li et al. designed targeted delivery of *quercetin* by biotinylated mixed micelles and demonstrated a high accumulation of *quercetin*-loaded mixed micelles at the tumor site and showed good anticancer activity in the mouse model of NSCLC [26]. The antitumor functions of the other three bioactive compounds are also found in documented reports of lung cancer or other cancers. Yao et al. demonstrated that *rhamnazin* may exert a therapeutic effect on pulmonary fibrosis by alleviating inflammation, oxidation, and collagen deposition via the TGF-*β*/Smad axis [27]. The antitumor effects of *rhamnazin* were also proved in hepatocellular carcinoma [28]. Wahyuni et al. thought *spinasterol* might have activity against cancer cells in triple-negative breast cancer [29]. Ravikumar et al. reported the antiproliferative and proapoptotic activities of *spinasterol* [30]. However, at present, *isofucosterol* is still rarely reported for its anti-obesity effect rather than its antitumor effect [31].

Three candidate targets with higher degree values in the core PPI network, MYC, ESR1, and HIF1A, were subjected to further molecular docking and analysis, and it was revealed that the three core targets had good affinity with the active compounds of *G. pentaphyllum*, referring to *quercetin* and MYC, *rhamnazin* and ESR1, and *quercetin* and HIF1A. c-Myc regulates multiple genes, which are associated with cell proliferation in many cancers, including NSCLC [32]. Guo et al. demonstrated *quercetin* notably repressed cancer cell proliferation by downregulating c-Myc expression in pancreatic ductal adenocarcinoma [33]. Chen et al. demonstrated *quercetin* could block the Akt/mTOR/c-Myc axis to inhibit the epithelial-mesenchymal transition of cancer cells [34]. *Quercetin* induces mesenchymal-to-epithelial transition by changing the nuclear localization of *β*-catenin and regulating *β*-catenin target genes, including c-Myc in triple-negative breast cancer [35]. In addition to MYC, we also found a stable binding with *quercetin* and HIF1A. The overexpression of HIF1A was found to predict poor survival in lung cancer [36]. Hassan et al. found that *quercetin* could enhance the cytotoxic activity of gemcitabine or doxorubicin on cancer cells by inhibiting HIF1A expression [37]. Tumova et al. treated human umbilical vein endothelial cells with *quercetin* to modulate glucose uptake/metabolism by affecting the stability of HIF1*α* [38]. Fulvestrant, as an estrogen receptor antagonist, was demonstrated to repress the epithelial-mesenchymal transition process of lung cancer cells, reducing tumor resistance to the cytotoxic effect of antigen-specific T cells and natural killer effector cells [39], suggesting that the contribution of ESR1 expression on lung cancer progression. The mechanism of *rhamnazin* and ESR1 interaction in experimental models of lung cancer cells is not investigated in reported studies, which may be required for further profound functional validation. The importance of network pharmacology has been emphasized in medical research [40].

When interpreting our results, several limitations should be noted. First, the molecular mechanism by which *G. pentaphyllum* treats NSCLC is not completely characterized as the public databases we used in the study have been updated continuously. Second, only three key genes received molecular docking and a lack of functional studies may weaken the reliability of the clinical translation. Third, experimental validation in vivo and in vitro focusing on the suppressive effects of two potential active compounds of G. pentaphyllum, quercetin and rhamnazin, on NSCLC cells as well as the expressions of MYC, ESR1, and HIF1A is warranted to improve the preliminary nature of the study.

## 5. Conclusions

In conclusion, our study demonstrates that *G. pentaphyllum*, especially its main active compounds, *quercetin* and *rhamnazin*, may exert therapeutic effects on NSCLC through the modulation of multiple targets, such as MYC, ESR1, and HIF1A. The present work also supports that the network pharmacology prediction method with molecular docking verification may provide a preliminary but systemic exploration focusing on the pharmacokinetic properties and mechanism of TCM in human diseases, offering opportunities to develop micelles for targeted delivery of TCM to tumor sites.

## Figures and Tables

**Figure 1:** Venn intersection analysis by R software showed there were 69 overlapping target genes of NSCLC and *G. pentaphyllum*.

**Figure 2:** Disease-target-compound network based on 8 bioactive compounds and 69 common targets. A red node represents disease, green nodes represent bioactive compounds of G pentaphyllum, and nodes in the outer ring represent common targets.

**Figure 3:** PPI network construction for disease-drug common targets (a) and their degree values (b) (here only listed targets with degree value more than 20).

**Figure 4:** Top 10 GO terms significantly enriched by disease-drug common targets at the levels of BP, CC, and MF (a) and KEGG pathways significantly enriched by disease-drug common targets (b). Larger circles reflect more enriched genes, and bluer indicates smaller *p* values.

**Figure 5:** Docking analysis of *quercetin* and MYC (a), *rhamnazin* and ESR1 (b), *quercetin* and HIF1A (c).

**Table 1:** The active ingredients of *G. pentaphyllum* with OB ≥ 30% concomitant with DL ≥ 0.18 in the TCMSP database.

Molecule ID	Molecule name	OB (%)	DL
MOL000338	3′-methyleriodictyol	51.61	0.27
MOL000351	Rhamnazin	47.14	0.34
MOL000359	Sitosterol	36.91	0.75
MOL004350	Ruvoside_qt	36.12	0.76
MOL004355	Spinasterol	42.98	0.76
MOL005438	Campesterol	37.58	0.71
MOL005440	Isofucosterol	43.78	0.76
MOL007475	Ginsenoside f2	36.43	0.25
MOL000953	CLR	37.87	0.68
MOL000098	Quercetin	46.43	0.28
MOL009855	(24S)-ethylcholesta-5,22,25-trans-3beta-ol	46.91	0.76
MOL009867	4*α*,14*α*-dimethyl-5*α*-ergosta-7,9(11),24(28)-trien-3*β*-ol	46.29	0.76
MOL009877	Cucurbita-5,24-dienol	44.02	0.74
MOL009878	Cyclobuxine	84.48	0.70
MOL009888	Gypenoside XXXVI_qt	37.85	0.78
MOL009928	Gypenoside LXXIV	34.21	0.24
MOL009929	Gypenoside LXXIX	37.75	0.25
MOL009938	Gypenoside XII	36.43	0.25
MOL009943	Gypenoside XL	30.89	0.21
MOL009969	Gypenoside XXXV_qt	37.73	0.78
MOL009971	Gypenoside XXVII_qt	30.21	0.74
MOL009973	Gypenoside XXVIII_qt	32.08	0.74
MOL009976	Gypenoside XXXII	34.24	0.25
MOL009986	Gypentonoside A_qt	36.13	0.80

## Data Availability

The data used to support the findings of this study are included within the article.
